# Pyrene-Phosphonate Conjugate: Aggregation-Induced Enhanced Emission, and Selective Fe^3+^ Ions Sensing Properties

This article has been retracted.

**DOI:** 10.3390/molecules22091417

**Published:** 2017-08-29

**Authors:** Sachin D. Padghan, Rajesh S. Bhosale, Sidhanath V. Bhosale, Frank Antolasic, Mohammad Al Kobaisi, Sheshanath V. Bhosale

**Affiliations:** 1 Polymers and Functional Materials Division, CSIR-Indian Institute of Chemical Technology, Hyderabad 500007, Telangana, India; padghansachu@gmail.com (S.D.P.); sidhanath.bhosale@gmail.com (S.V.B.); 2 School of Science, Royal Melbourne Institute of Technology University, GPO Box 2476, Melbourne, VIC 3001, Australia; m.alkobaisi@gmail.com (M.A.K.); frank.antolasic@rmit.edu.au (F.A.)

**Keywords:** pyrene-phosphonate, AIEE, optical and colorimetric, fluorescence, sensor of Fe^3+^ ions

## Abstract

A new pyrene-phosphonate colorimetric receptor **1** has been designed and synthesized in a one-step process via amide bond formation between pyrene butyric acid chloride and phosphonate-appended aniline. The pyrene-phosphonate receptor **1** showed aggregation-induced enhanced emission (AIEE) properties in water/acetonitrile (ACN) solutions. Dynamic light scattering (DLS) characterization revealed that the aggregates of receptor **1** at 80% water fraction have an average size of ≈142 nm. Field emission scanning electron microscopy (FE-SEM) analysis confirmed the formation of spherical aggregates upon solvent evaporation. The sensing properties of receptor **1** were investigated by UV-vis, fluorescence emission spectroscopy, and other optical methods. Among the tested metal ions, receptor **1** is capable of recognizing the Fe^3+^ ion selectively. The changes in spectral measurements were explained on the basis of complex formation. The composition of receptor **1** and Fe^3+^ ions was determined by using Job’s plot and found to be 1:1. The receptor **1**–Fe^3**+**^ complex showed a reversible UV-vis response in the presence of EDTA.

## 1. Introduction

Iron is an important element present in the earth’s crust and plays an important role in biochemical process [1,2]. For example, the balance of Fe^3+^ ion has significant effects on human health and various physiological functions [3,4,5]. Fe^3+^ ion acts as a cofactor in various enzymatic reactions in biological systems [6]. Iron deficiency causes low oxygen delivery to cells, low blood pressure, and immune deficiency, whereas its excess causes damage of lipids, nucleic acids, and proteins [7,8,9,10,11]. Alzheimer’s, Huntington’s, and Parkinson’s diseases are induced due to cellular toxicity caused by iron ions [12,13,14].

Aggregation-induced enhanced emission (AIEE) probes have been applied to monitor metal ions in many biological and environmental systems [15,16,17,18,19]. The development of AIEE probes for the detection of metal ions has also become an exciting research field [20,21]. The fabrication of such probes with synthetic ease, especially for important ions such as Fe^3+^, with the required sensitivity and selectivity is an important task that can enrich the toolbox of analytical chemistry in complex systems. This is in addition to the classical analytical methods with sophisticated instruments such as atomic absorption spectroscopy, inductively coupled plasma mass spectroscopy, and inductively coupled plasma-atomic emission spectrometry and cyclic voltammetry for the detection of Fe^3+^ ions [22,23,24,25]. Recently, several colorimetric and fluorescent methods were developed for the selective and sensitive detection of Fe^3+^ ions [26,27,28,29,30,31,32,33,34,35,36].

In this study, we report the design, synthesis, and characterization of the pyrene-phosphonate receptor **1**. This compound acts as a selective indicator toward Fe^3+^ ions. It also exhibits aggregation-induced enhanced emission (AIEE) properties and can be applied for selective visualization towards Fe^3+^ ions in the presence of a range of metal ions. To our knowledge, this is the first report on the colorimetric and fluorescence recognition of Fe^3+^ ions via complexation with biologically benign phosphonate functionality.

## 2. Results and Discussion

### 2.1. Design Strategy, Synthesis, and Characterization

Pyrene is a well-known organic florescent compound with environment-responsive vibrational fluorescence structures, a singlet long excited lifetime, and the ability to form excimers. Here, we used pyrene chromophore to design receptor **1**. Taking into account its properties, we conjugated pyrene chromophores with bisphosphonate phenyl rings. Receptor **1** was synthesized in a one-step amide bond formation between pyrene butyric acid chloride and phosphonate-appended aniline, as shown in Scheme 1. The obtained product was fully characterized using ^1^H-NMR, ^13^C-NMR, FT-IR, high-resolution mass spectrometry (HRMS), and electrospray ionisation mass spectrometry (ESI-MS).

### 2.2. A Naked Eye Detection of Metal Ions

In order to investigate the sensing properties of receptor **1** towards metal ions, it was co-solubilized with various metal ions such as Ag^+^, Al^3+^, Ba^2+^, Ca^2+^, Cd^2+^,Co^2+^, Cr^3+^, Cu^2+^, Hg^2+^, Fe^3+^, In^3+^, Mg^2+^, Mn^2+^,Ni^2+^, Pb^2+^, and Zn^2+^ in ACN:H_2_O (1:1). The results were monitored by observing the color change of receptor **1** with a naked eye upon complexation with the metal ions (Figure 1). The addition of per chlorate salt of Fe^3+^ into the solution of receptor **1** resulted in color changes from colorless to pale yellow. However, no color change of receptor **1** solution was observed with any of the other competitive metal ions mentioned above (Figure 1a). This indicated that Fe^3+^ ions interact with the phosphonate group of receptor **1** specifically, differently than with other metal ions on the electronic level [37]. The change in color of receptor **1** solution upon the addition of Fe^3+^ ions was also studied under UV light irradiation at 365 nm (Figure 1b), which showed a reduced blue fluorescence in the presence of Fe^3+^ ions in comparison to fluorescence in the presence of all other cations studied here. This fluorescent color change of receptor **1** was not observed with other competitive metal ions, indicating a selectivity towards Fe^3+^ ions.

### 2.3. Optical Sensing

The UV-vis absorption properties of receptor **1** were investigated in an ACN/H_2_O solution. Receptor **1** absorbance spectrum showed peaks at 240 nm, 270 nm, 280 nm, 337 nm, and 353 nm (Figure 2). Upon the addition of various metal ions such as Ag^+^, Al^3+^, Ba^2+^, Ca^2+^, Cd^2+^, Co^2+^, Cr^3+^, Cu^2+^, Hg^2+^, In^3+^, Mg^2+^, Mn^2+^, Ni^2+^, Pb^2+^, and Zn^2+^ in their perchlorate form to the receptor **1** solution showed negligible effect on the peaks intensity and position (Figure 2), whereas the addition of Fe^3+^ metal ions exhibited a hyperchromic shift in the spectrum of receptor **1**. Furthermore, we performed the systematic titration of Fe^3+^ with receptor **1**, as shown in Figure 2b; the increasing ratio of Fe^3+^ to receptor **1** resulted in a linear increase in the intensity of absorption peaks at 240 nm, 270 nm, 280 nm, 337 nm, and 353 nm. This titration also showed a hyperchromic shift in peak position, which was not observed for other metal ions.

### 2.4. Fluorescence Sensing

Fluorescence spectroscopy was employed to obtain detailed insight into the sensing properties of **1** towards various metal ions (Figure 3a). The fluorescence emission spectra of receptor **1** displays two peaks at 384 nm and 420 nm (λ_ex_ = 280 nm). The addition of competitive metal ions such as Ag^+^, Al^3+^, Ba^2+^, Ca^2+^,Cd^2+^,Co^2+^, Cr^3+^, Cu^2+^, Hg^2+^, In^3+^, Mg^2+^, Mn^2+^, Ni^2+^, Pb^2+^, and Zn^2+^ to receptor **1** showed negligible effect on the fluorescence emission characteristics of **1** (Figure 3a and Figure S1). On the other hand, the titration of receptor **1** with Fe^3+^ showed a decrease in fluorescence emission intensity. Figure 3b displays the linear decrease in the emission intensity of **1** at 384 nm and 420 nm with the increasing Fe^3+^ concentration.

This phenomenon can be qualitatively attributed to the effect of complexation on the charge transfer process from the phenyl phosphonate moiety to the pyrene fluorophore in the molecular structure. In the free ligand, charge transfer can occur freely between these two moieties, resulting in a weak florescence which can be enhance with aggregation and the restriction of the thermal relaxation via conformational rotations in the free alkyl linking chain [38,39].

This relaxation is less affected by cations with low charge density, while Fe^3+^ can significantly affect the electronic and the conformational structure of **1** in the complex (see Figure 4a). Therefore, this charge transfer is significantly reduced due to the increase in the ionization/oxidation potential of the phenyl phosphonate moiety. The suppression of the charge transfer between the acceptor and the donor moieties of **1** is also affected, due to the existence of the Fe^2+^ oxidation state, which causes the Fe^3+^ metal ion to become the new acceptor in the complex structure.

The energy modeling of the complex using Gaussian 09 at UB3LYP/SDD and sextet spin multiplicity level of theory showed that the HOMO (185) is concentrated on the pyrene moiety and the LUMO is concentrated on the phenyl phosphonate–Fe^3+^ of the complex moiety. This confirms the charge transfer to the cation center producing the Fe^2+^ oxidation state of the iron cation (see Figure 4b) [40].

We also examined the changes in UV-vis absorption and fluorescence emission of receptor **1** upon the addition of Fe^2+^ ions, and found negligible changes, as shown in Figure S2a,b, respectively. Thus, it can be concluded that receptor **1** has higher selectivity towards Fe^3+^ ions. The results obtained by colorimetric and UV-vis experiments were supported by the fluorescence emission studies of receptor **1** towards Fe^3+^ ion addition.

The linear relationship was obtained. The Benesi-Hildebrand equation (Figure S3) was used to calculate the association constant (*K_a_*) of receptor **1** for Fe^3+^ ions, which was found to be 5 × 10^13^ M^−1^. Moreover, Job’s plot (Figure S4) was employed to determine the stoichiometry of the complex between receptor **1** and Fe^3+^ ions, which was confirmed to be 1:1. The detection of limit was evaluated in order to determine the practical applicability of receptor **1**. The equation 3*S*/*ρ* was employed for to calculate the limit of detection, where *S* is the standard deviation of three blank measurements and *ρ* is the slope between the emission intensity versus the concentration of the receptor. The limit of detection was calculated using the linear relationship between the fluorescence emission at 384 nm and the concentration of Fe^3+^ ions (Figure S5). Receptor **1** has a limit of detection of 0.99 μM for Fe^3+^ ions.

### 2.5. Competitive Experiments

We investigated the competitive metal ion binding studies of receptor **1** towards selective sensing of Fe^3+^ ions in the presence of interfering metal ions (10 equiv.) such as Ag^+^, Al^3+^, Ba^2+^, Ca^2+^, Cd^2+^, Co^2+^, Cr^3+^, Cu^2+^, Hg^2+^, In^3+^, Mg^2+^, Mn^2+^, Ni^2+^, Pb^2+^, and Zn^2+^. The fluorescence emission experiments were performed, and the results are depicted in Figure 5. The presence of interfering metal ions did not show any significant change in the emission spectrum, as obtained by the addition of only Fe^3+^ ions to receptor **1**. Thus, these experiments clearly showed the non-interference of the tested metal ions on the selective detection of Fe^3+^ ions by receptor **1**.

The employed colorimetric, UV-vis absorption, and fluorescence emission spectroscopic techniques confirmed that receptor **1** exhibits selectivity towards Fe^3+^ ions. To confirm the nature of the complex formation between receptor **1** and Fe^3+^ ions, the Fourier transform infrared (FT-IR) spectrum of receptor **1** was recorded in the absence and presence of Fe^3+^ ions (Figure 6). The IR spectrum of receptor **1** shows P=O bond stretching vibration at 1240 cm^−1^ and P-O-C (alkyl) bond vibrations at 1053 cm^−1^ and 1024 cm^−1^ of the phosphonate ester groups of the receptor [41]. After the complexation between receptor **1** and Fe^3+^ ions, the band at 1240 cm^−1^ shifted to 1249 cm^−1^ with decreasing intensity. The intensity of bands at 1053 cm^−1^ and 1024 cm^−1^ were also notably decreased after complexation. Based on the IR study, we can hypothesize that the two phosphonate ester groups of receptor **1** coordinate with Fe^3+^ ions in the complex formation.

There is an indication of an electron transfer occurring from the pyrene to Fe^3+^. Since the ratio between ligand **1** and Fe^3+^ is 1:1, to complete the coordinates there is a good chance that the metal ion is sandwiched between the phosphonate groups and the aromatic pyrene [42,43].

Fe^3+^ + Ligand **1** → Fe^2+^ + Ligand **1** (1+) (1)

This electron transfer (or partial charge transfer) can affect the optical characteristics of the complex. Metal ions with only one oxidation state or low charge density would not be able to induce this possible charge transfer event.

For practical applications, reversibility is an important aspect in the chemical receptor. Receptor **1** is sensitive towards the detection of Fe^3+^ ions. It is well known that ethylenediaminetetraacetic acid (EDTA) binds to Fe^3+^. We have used EDTA to examine the reversibility of the **1**–Fe^3+^ complex. The gradual addition of EDTA to the **1**–Fe^3+^ complex resulted in a significant increase in the fluorescence emission peak intensity at 384 nm and 420 nm (Figure 7). These experiments confirm a return of the maximum emission peak intensity to its original state. Thus, fluorescence emission spectroscopy experiments support the reversibility of receptor **1** towards Fe^3+^ ions.

### 2.6. Aggregation-Induced Enhanced Emission (AIEE) Phenomenon

The selectivity of the probe towards cations was incredibly affected due to AIEE properties [44,45]. Therefore, we examined the emission response of **1** in the direction of AIEE. As shown in Figure 8, the emission experiments were recorded for **1** upon the incremental addition of water fraction from 0% to 95% in ACN. The increase in fluorescence emission peaks at 384 nm and 420 nm (λ_ex_ = 280 nm) with respect to *f_w_* (0–80%) was observed. The emission intensity starts to rise at *f_w_* > 10% and continues to increase until *f_w_* 80%, at which point the solvating influence of the mixture is worsened to such an extent that the molecules start to aggregate. These results clearly indicate that the probe **1** showed AIEE properties in *f_w_* = 80% upon aggregation. Furthermore, we examined the quantum yield (*Φ_f_*) of probe **1**. The initial quantum yield of **1** in a dissolved state in acetonitrile i.e., at 0% *f_w_* (*Φ_f_* = 1.9), which was increased by ~6-fold to the maximum value at 80% *f_w_* (*Φ_f_* = 11.7). In colorimetric response, a strong blue emission was observed under UV light at 365 nm (Figure S6). This result strongly supports the AIEE of probe **1** in H_2_O (0–80%). The further addition of water (*f_w_* > 80%) led to the downfall of the emission, which is due to the precipitate formation; the photoluminescence (PL) intensity decreases to some extent as both water and acetonitrile are hydrophilic solvents and only the smaller aggregates in the suspension contributed to the emission, as indicated by the data shown in the inset of Figure 8. However, there was not much influence observed on the emission efficiency; at *f_w_* 80% and 90%, *Φ* is about 11.7% and 7.9%, respectively (see ESI Table S1) [46]. Such emission behavior is referred to as the AIEE effect, thus, compound 1 is AIE active. This was also confirmed by dynamic light scattering, showing that ~90% of the water content’s average hydrodynamic diameter increased to 175 nm (ESI Figure S7).

### 2.7. Visualization of Aggregates by FE-SEM Analysis and Dynamic Light Scattering (DLS) Analysis

To gain further insight and to further investigate the mode of aggregation of compound **1** from 80% water/CH_3_CN, field emission scanning electron microscopy (FE-SEM) and dynamic light scattering (DLS) were employed. Particular aggregates were produced upon water/CH_3_CN evaporation of **1** (10^−5^ M) by drop-casting on a silicon wafer substrate. SEM analysis clearly shows that compound **1** produced spherical particles with varying sizes of ~150–300 nm (Figure 9a). Furthermore, DLS analysis shows a hydrodynamic diameter with an average size of ≈142 nm (Figure 9b), which is indicative of the dynamic interaction of the molecules in the solution. We also examined the effect of different water content in ACN solution of **1**. The addition of water to acetonitrile solution of **1** to form a volume ratio of 60%, 70%, and 90%, showed an increase in the average hydrodynamic diameter up to 98 nm, 137 nm, and 175 nm, respectively (Figure S7). We speculate that this was due to the increase in the water content, which might cause larger sizes of aggregates.

## 3. Experimental Section 

### 3.1. Materials and Instruments

All chemicals for synthesis were purchased from Sigma Aldrich (Bengaluru, Karnataka, India) and were used without further purification, unless otherwise specified. Freshly prepared deionized water was used for sample preparation. The stock solutions of the metal ions were prepared from their perchlorate salts. ^1^H-NMR spectra were recorded on Bruker AVANCE 500 MHz and ^13^C-NMR 125 MHz NMR spectrometers (Rheinstetten, Germany), using tetramethylsilane (TMS) as the internal standard and CDCl_3_-*d* as the solvent. Mass spectrometric data were obtained by the positive electron spray ionization (ESI-MS) technique on an Agilent Technologies 1100 Series (Agilent Chemistation Software, Agilent Technologies, Inc., Santa Clara, CA, USA) mass spectrometer. High-resolution mass spectra (HRMS) were obtained by using ESIQTOF mass spectrometry. FTIR spectra were recorded on a Perkin Elmer FT-IR 400 spectrometer (Arcade, New York, USA). UV-vis absorption spectra were recorded by a UV-vis-1800 Shimadzu (Tokyo, Japan) spectrophotometer. Fluorescence emission spectra were measured on an RF-6000 (Shimadzu, Tokyo, Japan) spectrofluorophotometer.

### 3.2. Naked-Eye Colorimetric Response

The anion solutions were added to a solution of probe **1** (25 μM) in an ACN:water (1:1; *v*/*v*) solvent mixture. With the addition of anion solutions (3 equiv.) to receptor **1,** the image was recorded with a well-resolved camera at room temperature.

### 3.3. UV-Vis Absorption Spectroscopic

Probe **1** was dissolved in an ACN:water (1:1; *v*/*v*) solvent mixture with c ≈ 1.0 × 10^−5^ M corresponding to the maximum absorbance in the range ≈0.1 to 0.4 for the UV experiments. The solution of the probe **1** was placed in a quartz cuvette (*Ɩ* = 1 cm, V_0_ = 3 mL) followed by the addition of various metal ion solutions (c ≈ 1 mM). UV-vis spectrum was recorded at room temperature.

### 3.4. Fluorescence Spectroscopic

To a solution of **1** (1.0 × 10^−5^ M) in an ACN:water (1:1; *v*/*v*) mixture, the various metal ion solutions were added. Emission spectra were recorded with an excitation wavelength of (λ_ex_ = 280 nm) with each addition at room temperature.

### 3.5. Reversible Experimental with EDTA

EDTA solution in an ACN:H_2_O (1:1, *v*/*v*) mixture was added to the solution of **1**–Fe^3+^ complex in a 3 mL quartz cuvette. The gradual addition of EDTA to the **1**–Fe^3+^ complex solution was monitored using fluorescence spectroscopy. The fluorescence emission was monitored upon excitation at wavelength 280 nm.

### 3.6. FE-SEM Measurements

The silicon wafer was first cleaned by acetone, followed by ethanol and then Milli Q water. SEM samples were prepared by solvent evaporation on a silicon wafer and then sputter-coated with gold for 10 s at 0.016 mA Ar plasma (SPI, West Chester, PA, USA) for SEM imaging using an FEI Nova NanoSEM (Hillsboro, OH, USA) operating at high vacuum.

### 3.7. DLS Analysis

DLS measurements were conducted using Brookhaven Instrument Corp. (Holtsville, NY, USA), 90Plus Particle Size equipped with a He-Ne laser (632.8 nm, 35 mW) and quartz cuvette.

### 3.8. Synthesis and Characterization of Target Molecules

#### 3.8.1. Synthesis of 1-Pyrene Butyric Acid Chloride

1-Pyrene butyric acid (700 mg, 2.42 mol) in 25 mL CH_2_Cl_2_ and thionyl chloride (4.26 mL, 58.51 mol) was added under nitrogen conditions, and the reaction mixture was refluxed for 6 h at 80 °C. Excess thionyl chloride and CH_2_Cl_2_ was removed under reduced pressure. A blackish sticky product was formed, which further used for next step without further purification.

#### 3.8.2. Synthesis of Pyrene Phosphonate

Pyrenebutyric acid chloride (500 mg, 1.63 mmol) in 30 mL of CH_2_Cl_2_ was added to the phosphonate-appended aniline (700 mg, 1.52 mmol) at 0 °C and vigorously stirred. Triethyl amine (1 mL) was added to the reaction mixture at 0 °C. The reaction mixture was further stirred overnight at room temperature. The reaction mixture was then poured in sodium bicarbonate solution with stirring and extracted using CH_2_Cl_2_. The organic layer was washed with 0.1 N HCL and brine solution. The solvent was evaporated under reduced pressure. The obtained product was purified by flash column chromatography on silica (eluting with 1:99 DCM: CH_3_OH) to afford pure compound **1**. FT-IR (KBr, *v* cm^−1^): 515, 711, 783, 846, 965, 1027, 1053, 1240, 1437, 1463, 1563, 1606, 1684, 2929, 2982, 3272 and 3433. ^1^H-NMR (500 MHz, CDCl_3_) δ: 1.22 (t, *J* = 7.01 Hz, 12H), 2.24 (m, 2H), 2.46 (t, *J* = 7.01 Hz, 2H), 3.05 (s, 4H), 3.39 (t, *J* = 7.17 Hz, 2H), 4.01 (m, 8H), 6.92 (s, 1H), 7.40 (s, 2H), 8.01 (m, 10H). ^13^C-NMR (125 MHz, CDCl_3_) δ: 16.3, 27.05, 32.8, 33.9, 36.6, 62.1, 119.4, 128.1, 129.3, 130.2, 132.3, 135.7, 136.4, 138.7, 171.05; ^31^P NMR (200 MHz, CDCl_3_) δ: 277.5; ESI-MS (*m*/*z* %): 665 (100) [M + H] ^+^. HRMS: calculated for C_36_ H_44_ O_7_ N P = 664.26052, found [M^+^] = 664.25875.

## 4. Conclusions

In conclusion, we have shown the synthesis and utility of a new pyrene-based receptor **1** as a colorimetric and fluorescence chemosensor for the selective detection of Fe^3+^ ions. Receptor **1** showed AIEE characteristics upon the addition of water (0–80%) in ACN. The fluorescence switch-off mechanism was involved. The sensing selectivity of receptor **1** was established by means of UV-vis absorption and fluorescence spectroscopy-based experiments. It is worth mentioning that the sensing capability of receptor **1** also can be established by the naked-eye detection method. Interestingly, compound **1** gives the AIEE effect upon aggregation as a defined spherical particle from 80% water/acetonitrile solution. Thus, the present method of Fe^3+^ detection opens up the possibility of using this phosphonate-appended pyrene probe for biological applications, and work toward this direction is in progress in our laboratory and will be reported in due course.

## Figures and Tables

**Scheme 1:** Synthesis of phosphonate-appended pyrene receptor **1**.

**Figure 1:** (**a**) Color of receptor **1** with different metal ions, (**b**) fluorescence of receptor **1** under UV irradiation (λ_ex_ = 365 nm) in the presence of various metal ions.

**Figure 2:** (**a**) UV-vis absorption spectra of receptor **1** (c = 1.0 × 10^−5^ M) upon the addition of metal ions (10 equiv.); (**b**) Receptor **1**–Fe^3+^ ion at 0–10 equiv. Fe^3+^ ratios where receptor **1** c = 1.0 × 10^−5^ M; Inset-linear plot of intensity vs. concentration at 279-nm wavelength.

**Figure 3:** (**a**) Fluorescence spectra of receptor **1** (c = 1.0 × 10^−5^ M) upon the addition of various metal ions (10 equiv.); excitation wavelength: 280 nm. (**b**) Fe^3+^ concentration-dependent changes in the fluorescence spectra of **1** (c = 1.0 × 10^−5^ M) upon the addition of Fe^3+^ ions (0–10 equiv.); excitation wavelength: 280 nm.

**Figure 4:** (**a**) Schematic representation of the fluorophore emission of receptor **1** in the presence and absence of Fe^3+^ cations, showing the excited state relaxation restriction in **1** + Fe^3+^ complex; (**b**) The electronic structure of the **1** + Fe^3+^ complex as calculated using UB3LYP/SDD and sextet spin multiplicity level of theory.

**Figure 5:** Metal-ion selectivity of receptor **1** towards Fe^3+^ ions (10 μM) in the presence of competitive ions (10 μM): 1 (receptor **1**); 2 (**1** + Fe^3+^); 3 (**1** + Ag^+^ + Fe^3+^); 4 (**1** + Al^3+^ + Fe^3+^); 5 (**1** + Ba^2+^ + Fe^3+^); 6 (**1** + Ca^2+^ + Fe^3+^); 7 (**1** + Cd^2+^ + Fe^3+^); 8 (**1** + Co^2+^ + Fe^3+^); 9 (**1** + Cr^3+^ + Fe^3+^); 10 (**1** + Cu^2+^ + Fe^3+^); 11 (**1** + Hg^2+^ + Fe^3+^); 12 (**1** + In^3+^ + Fe^3+^); 13 (**1** + Mg^2+^ + Fe^3+^) 14 (**1** + Mn^2+^ + Fe^3+^); 15 (**1** + Ni^2+^ + Fe^3+^); 16 (**1** + Pb^2+^ + Fe^3+^); 17 (**1** + Zn^2+^ + Fe^3+^).

**Figure 6:** Comparison between the FT-IR spectral data of receptor **1** and the **1**–Fe^3+^ ion complex.

**Figure 7:** Fluorescence intensity changes of **1** upon the addition of Fe^3+^ and the demetalation (removal of Fe^3+^) by the addition of EDTA in ACN:H_2_O (1:1, *v*/*v*).

**Figure 8:** Aggregation-induced emission enhancement of **1** upon the incremental addition of water from 0% to 95% to ACN (λ_ex_ = 280 nm); Inset: change in intensity with respect to water fraction.

**Figure 9:** (**a**) Field emission scanning electron micrographs (FE-SEM) of the spherical aggregate of **1** (10^−5^ M) upon solvent evaporation on a silicon wafer; (**b**) Average hydrodynamic diameter of 80% water/acetonitrile aggregates and the size measured using a dynamic light scattering (DLS) particle size analyzer.

## Supplementary Materials

Supplementary materials are available online.

## References

[1] Cairo G., Pietrangelo A. (2000). Iron regulatory proteins in pathobiology. Biochem. J..

[2] Touati D. (2000). Iron and oxidative stress in bacteria. Arch. Biochem. Biophys..

[3] Weizman H., Ardon O., Mester B., Libman J., Dwir O., Hadar Y., Chen Y., Shanzer A. (1996). Fluorescently-labeled ferrichrome analogs as probes for receptor-mediated, microbial iron uptake. J. Am. Chem. Soc..

[4] D’Autreaux B., Tucker N.P., Dixon R., Spiro S. (2005). A non-haem iron centre in the transcription factor norr senses nitric oxide. Nature.

[5] Lee J.-W., Helmann J.D. (2006). The perr transcription factor senses H_2_O_2_ by metal-catalysed histidine oxidation. Nature.

[6] Kaim W., Schwederski B., Klein A. (2013). Bioinorganic Chemistry: Inorganic Elements in the Chemistry of Life: An Introduction and Guide.

[7] Crown J.A. (1997). Inorganic Biochemistry: An Introduction.

[8] Haas J.D., Brownlie T. (2001). Iron deficiency and reduced work capacity: A critical review of the research to determine a causal relationship. J. Nutr..

[9] Halliwell B., Gutteridge J.M.C. (1990). Role of free radicals and catalytic metal ions in human disease: An overview. Methods Enzymol..

[10] Halliwell B., Gutteridge J.M.C. (1992). Biologically relevant metal ion-dependent hydroxyl radical generation an update. FEBS Lett..

[11] Halliwell B., Gutteridge J.M.C. (1999). Free Radicals in Biology and Medicine.

[12] Crichton R.R., Dexter D.T., Ward R.J. (2008). Metal based neurodegenerative diseases—From molecular mechanisms to therapeutic strategies. Coord. Chem. Rev..

[13] Dornelles A.S., Garcia V.A., de Lima M.N.M., Vedana G., Alcalde L.A., Bogo M.R., Schröder N. (2010). Mrna expression of proteins involved in iron homeostasis in brain regions is altered by age and by iron overloading in the neonatal period. Neurochem. Res..

[14] Ong W.-Y., Farooqui A.A. (2005). Iron, neuroinflammation, and alzheimer’s disease. J. Alzheimers Dis..

[15] Hong Y., Lam J.W.Y., Tang B.Z. (2011). Aggregation-induced emission. Chem. Soc. Rev..

[16] Yuan Y., Zhang C.-J., Gao M., Zhang R., Tang B.Z., Liu B. (2015). Specific light-up bioprobe with aggregation-induced emission and activatable photoactivity for the targeted and image-guided photodynamic ablation of cancer cells. Angew. Chem. Int. Ed..

[17] Ding D., Li K., Liu B., Tang B.Z. (2013). Bioprobes based on aie fluorogens. Acc. Chem. Res..

[18] Liang J., Tang B.Z., Liu B. (2015). Specific light-up bioprobes based on aiegen conjugates. Chem. Soc. Rev..

[19] Hong Y., Meng L., Chen S., Leung C.W.T., Da L.-T., Faisal M., Silva D.-A., Liu J., Lam J.W.Y., Huang X. (2012). Monitoring and inhibition of insulin fibrillation by a small organic fluorogen with aggregation-induced emission characteristics. J. Am. Chem. Soc..

[20] Amendola V., Fabbrizzi L., Foti F., Licchelli M., Mangano C., Pallavicini P., Poggi A., Sacchi D., Taglietti A. (2006). Light-emitting molecular devices based on transition metals. Coord. Chem. Rev..

[21] Yang Y., Zhao Q., Feng W., Li F. (2013). Luminescent chemodosimeters for bioimaging. Chem. Rev..

[22] Andersen J.E.T. (2005). A novel method for the filterless preconcentration of iron. Analyst.

[23] Del Castillo Busto M.E., Montes-Bayón M., Blanco-González E., Meija J., Sanz-Medel A. (2005). Strategies to study human serum transferrin isoforms using integrated liquid chromatography icpms, maldi-tof, and esi-q-tof detection:  Application to chronic alcohol abuse. Anal. Chem..

[24] Pomazal K., Prohaska C., Steffan I., Reich G., Huber J.F. (1999). Determination of Cu, Fe, Mn, and Zn in blood fractions by sec-hplc-icp-aes coupling. Analyst.

[25] Van den Berg C.M.G. (2006). Chemical speciation of iron in seawater by cathodic stripping voltammetry with dihydroxynaphthalene. Anal. Chem..

[26] Sahoo S.K., Sharma D., Bera R.K., Crisponi G., Callan J.F. (2012). Iron(iii) selective molecular and supramolecular fluorescent probes. Chem. Soc. Rev..

[27] Carter K.P., Young A.M., Palmer A.E. (2014). Fluorescent sensors for measuring metal ions in living systems. Chem. Rev..

[28] Chung P.K., Liu S.-R., Wang H.-F., Wu S.-P. (2013). A pyrene-based highly selective turn-on fluorescent chemosensor for iron(iii) ions and its application in living cell imaging. J. Fluoresc..

[29] Mukherjee S., Talukder S. (2016). A reversible pyrene-based turn-on luminescent chemosensor for selective detection of Fe^3+^ in aqueous environment with logic gate application. J. Fluoresc..

[30] Weerasinghe A.J., Schmiesing C., Varaganti S., Ramakrishna G., Sinn E. (2010). Single- and multiphoton turn-on fluorescent Fe^3+^ sensors based on bis(rhodamine). J. Phys. Chem. B.

[31] Lim N.C., Pavlova S.V., Brückner C. (2009). Squaramide hydroxamate-based chemidosimeter responding to iron(iii) with a fluorescence intensity increase. Inorg. Chem..

[32] Xiang Y., Tong A. (2006). A new rhodamine-based chemosensor exhibiting selective Fe(iii)-amplified fluorescence. Org. Lett..

[33] Bricks J.L., Kovalchuk A., Trieflinger C., Nofz M., Büschel M., Tolmachev A.I., Daub J., Rurack K. (2005). On the development of sensor molecules that display Fe(iii)-amplified fluorescence. J. Am. Chem. Soc..

[34] Yang Z., She M., Yin B., Cui J., Zhang Y., Sun W., Li J., Shi Z. (2012). Three rhodamine-based “off-on” chemosensors with high selectivity and sensitivity for Fe^3+^ imaging in living cells. J. Org. Chem..

[35] Li N., Xu Q., Xia X., Wang L., Lu J., Wen X. (2009). A polymeric chemosensor for Fe^3+^ based on fluorescence quenching of polymer with quinoline derivative in the side chain. Mater. Chem. Phys..

[36] Xu M., Wu S., Zeng F., Yu C. (2010). Cyclodextrin supramolecular complex as a water-soluble ratiometric sensor for ferric ion sensing. Langmuir.

[37] Tolis E.I., Helliwell M., Langley S., Raftery J., Winpenny R.E.P. (2003). Synthesis and characterization of iron(iii) phosphonate cage complexes. Angew. Chem. Int. Ed..

[38] De Silva A.P., Gunaratne H.Q.N., Gunnlaugsson T., Huxley A.J.M., McCoy C.P., Rademacher J.T., Rice T.E. (1997). Signaling recognition events with fluorescent sensors and switches. Chem. Rev..

[39] Hayashita T., Yamauchi A., Tong A.-J., Lee J.C., Smith B.D., Teramae N. (2004). Design of supramolecular cyclodextrin complex sensors for ion and molecule recognition in water. J. Incl. Phenom. Macrocycl. Chem..

[40] Frisch M.J., Trucks G.W., Schlegel H.B., Scuseria G.E., Robb M.A., Cheeseman J.R., Scalmani G., Barone V., Petersson G.A., Nakatsuji H. (2016). Gaussian 09, Revision A.02.

[41] Alexandratos S.D., Zhu X. (2015). The role of polarizability in determining metal ion affinities in polymer-supported reagents: Monoprotic phosphates and the effect of hydrogen bonding. New J. Chem..

[42] Venkatesan P., Wu S.-P. (2015). A turn-on fluorescent pyrene-based chemosensor for Cu(ii) with live cell application. RSC Adv..

[43] D’Aléo A., Cecchetto E., De Cola L., Williams R. (2009). Metal ion enhanced charge transfer in a terpyridine-bis-pyrene system. Sensors.

[44] Shellaiah M., Simon T., Srinivasadesikan V., Lin C.-M., Sun K.W., Ko F.-H., Lin M.-C., Lin H.-C. (2016). Novel pyrene containing monomeric and dimeric supramolecular aiee active nano-probes utilized in selective “off-on” trivalent metal and highly acidic ph sensing with live cell applications. J. Mater. Chem. C.

[45] Shellaiah M., Wu Y.-H., Singh A., Ramakrishnam Raju M.V., Lin H.-C. (2013). Novel pyrene- and anthracene-based schiff base derivatives as Cu^2+^ and Fe^3+^ fluorescence turn-on sensors and for aggregation induced emissions. J. Mater. Chem. A.

[46] Rananaware A., La D.D., Bhosale S.V. (2015). Solvophobic control aggregation-induced emission of tetraphenylethene-substituted naphthalene diimide via intramolecular charge transfer. RSC Adv..

